RETRACTED

# Ribosome-Dependent ATPase Interacts with Conserved Membrane Protein in *Escherichia coli* to Modulate Protein Synthesis and Oxidative Phosphorylation

**DOI:** 10.1371/journal.pone.0018510

**Published:** 2011-04-27

**Authors:** Mohan Babu, Hiroyuki Aoki, Wasimul Q. Chowdhury, Alla Gagarinova, Chris Graham, Sadhna Phanse, Ben Laliberte, Noor Sunba, Matthew Jessulat, Ashkan Golshani, Andrew Emili, Jack F. Greenblatt, M. Clelia Ganoza

**Affiliations:** 1 Banting and Best Department of Medical Research, University of Toronto, Toronto, Ontario, Canada; 2 Department of Molecular Genetics, University of Toronto, Toronto, Ontario, Canada; 3 Department of Biology and Ottawa Institute of Systems Biology, Carleton University, Ottawa, Canada; University of Kent, United Kingdom

## Abstract

Elongation factor RbbA is required for ATP-dependent deacyl-tRNA release presumably after each peptide bond formation; however, there is no information about the cellular role. Proteomic analysis in *Escherichia coli* revealed that RbbA reciprocally co-purified with a conserved inner membrane protein of unknown function, YhjD. Both proteins are also physically associated with the 30S ribosome and with members of the lipopolysaccharide transport machinery. Genome-wide genetic screens of *rbbA* and *yhjD* deletion mutants revealed aggravating genetic interactions with mutants deficient in the electron transport chain. Cells lacking both *rbbA* and *yhjD* exhibited reduced cell division, respiration and global protein synthesis as well as increased sensitivity to antibiotics targeting the ETC and the accuracy of protein synthesis. Our results suggest that RbbA appears to function together with YhjD as part of a regulatory network that impacts bacterial oxidative phosphorylation and translation efficiency.

## Introduction

Protein synthesis on ribosomes requires GTPase and ATPase factors. During protein chain elongation, EF-Tu, a GTPase recruits the activated aminoacyl-tRNA to the ribosomal A-site. RbbA or Ribosome Bound ATPase, acts in conjunction with EF-Tu to poise the aminoacyl-tRNA on the ribosomal A-site [1]. After peptide bond formation by the peptidyl transferase, the growing peptide is bound to the tRNA in the A-site and the deacyl-tRNA to the P-site. Subsequently, EF-G, a ribosome-associated GTPase, promotes the translocation of the ribosome and the tRNAs one codon at a time relative to the mRNA in the 5′direction, transferring the newly formed peptidyl-tRNA to the P-site, the deacyl-tRNA to the E-site and exposing the ribosomal A-site to the next aminoacyl-tRNA [2].

The ribosome-dependent ATPase, RbbA in *Escherichia coli*, markedly stimulates synthesis in reconstituted extracts [3]. RbbA is encoded within its own operon by a gene non-essential for growth at neutral pH [4]. The amino acid sequence of RbbA reveals two ATP binding motifs, two Walker motifs that define most ABC transporters [1], one RNA-binding motif and six predicted transmembrane helices. Omission of RbbA (formerly W) arrests synthesis at the dipeptide stage and deacyl-tRNA remains bound to ribosomes. RbbA promotes release of deacyl-tRNA from ribosomes and ensuing synthesis [3] as well as stimulates ejection of deacyl-tRNA by accelerating binding of EF-Tu•GTP•aminoacyl-tRNA to ribosomes [1]. Indeed, chemical protection footprints indicate that RbbA binds directly to the ribosomal E-site [1]. The E-site is involved in deacyl-tRNA ejection, translocation and reading frame maintenance [5]. The ribosome and RbbA-dependent hydrolysis of ATP as well as the transfer of acylated aminoacyl-tRNAs is inhibited by the ATP analogue, AMPPpC, suggesting that the hydrolysis of ATP is indeed required during synthesis [6]. If, in fact, RbbA stimulates the ribosome-dependent hydrolysis of ATP after each peptide bond is formed upon release of each deacyl-tRNA, then the energy requirements for synthesis correspondingly increase. In this context, and considering the total metabolic, energy demand imposed by the translation process [7], it seems reasonable to assume that this process is associated with an energy source to rapidly replenish energy and maintain cellular viability.

RETRACTED

To gain insight into the cellular role of RbbA, we performed genome-wide physical and genetic interactions involving RbbA from *E. coli*. We found that RbbA bound to the membrane where it reciprocally co-purifies with an inner membrane (IM) protein of unknown function, YhjD. Both these tagged proteins physically interact with members of the lipopolysaccharide (LPS) transport pathway and localize to the 30S ribosomal subunits. Genome-wide genetic screens of *rbbA* and *yhjD* displayed aggravating interactions with members of the electron transport chain (ETC). Strains lacking *rbbA* and *yhjD* showed defects in growth, cell division, respiration and protein synthesis and increased sensitivity to chemical agents that block the ETC and to antibiotics affecting translational fidelity and translocation. Collectively, these and supporting data suggest that RbbA has a dual role in the cell, which, in conjunction with YhjD, links protein synthesis to several membrane processes including LPS transport and energy regeneration.

## Results

### RbbA Physically Associates with Protein Synthesis and Membrane Processes

To probe the cellular aspects of RbbA function, we performed an unbiased protein interaction screen to identify its physical interaction partners *in vivo*. Full-length RbbA was affinity-tagged at its C-terminal end by recombining a SPA (Sequential Peptide Affinity) cassette (consisting of a triple FLAG tag and a calmodulin binding peptide) into the chromosome [8]. SPA-tagged RbbA was extracted from the membranes of log-phase cultures in the absence of detergents as well as using three different mild non-ionic detergents [Triton X 100, DDM (n-dodecyl-β-D-maltopyranoside), and C_12_E_8_ (Octaethylene glycol monododecyl ether)] at 1% concentrations, following which the stably associated proteins were affinity-purified in two steps on anti-FLAG and calmodulin resins and then identified using tandem mass spectrometry (LCMS) and peptide mass fingerprinting (MALDI-TOF MS). Three purifications with different detergents were used [9] to optimize the solubilization and partly validate interacting proteins.

RETRACTED

Purification of RbbA in the detergent extracts detected a 91 kDa full-length RbbA, while the protein was not detected in purifications without detergents, suggesting that it is tightly bound to the membrane fraction (**Table S1**). The 91 kDa RbbA also occurs tightly bound to the ribosomes [10] because the conditions used to extract RbbA from the membranes were expected to disrupt ribosome structure and may thus not be seen in the detergent free-extract. To minimize potential non-specific interactions, we considered only proteins that co-purified with RbbA in at least two different detergents as *bona fide* interactors (**Table S1**). Using this stringent filtering criteria, we found RbbA bound to protein synthesis elongation factor EF-Tu (e.g. TufA and TufB), 30S (e.g. RpsE, RpsJ, RpsM, RpsN, RpsP, RpsS and RpsT) subunit ribosomal (r) proteins, to other cytoplasmic proteins involved in tRNA (e.g., CCA) and rRNA (e.g. Rng, RlmL) processing (**Text S1**) and with the release factor PrfA (**Table S1**). The endogenous affinity-tagged RbbA also co-purified efficiently with several energy regeneration (e.g. AceE, FdoH and FruR) and membrane (e.g. LolB, Trg, MrcB, SecD, WcaM, LptD) components (**Text S1**) including YhjD, a putative IM protein of unknown function with 5–6 transmembrane helices that had tentatively been implicated in lipid A precursor IV_A_ transport [11], [12] (**Table S1**).

Amongst the proteins that interact with RbbA, the putative non-essential IM protein YhjD was selected because it harbors an RNA binding (residues 60 to 65) and two ATP binding (residues 118 to 123 and 235–241) motifs in its amino acid sequence (**Figure S1**). The RNA binding motif in YhjD is homologous to RNase BN, which is involved in tRNA processing [SSDB (Sequence Similarity DataBase) motif result, data not shown]. Since RbbA and YhjD share these common motifs, we performed reciprocal affinity purification in the presence of three detergents using an endogenously expressed SPA-tagged YhjD strain and searched for physical interactions with other *E. coli* proteins and membrane functions as well its possible functional connection with RbbA in protein synthesis.

RETRACTED

The affinity-tagged YhjD specifically co-purified with RbbA in two different detergents (**Table S1**). Neither of these binding partners was detected in parallel purifications from an untagged negative control strain or from several hundred previously studied SPA-tagged bait proteins [13]. Additionally, the ectopically expressed hexahistidine (His_6_)- tagged RbbA, efficiently co-precipitated with YhjD in detergent extracts, but not with an untagged or other functionally unrelated tagged proteins (**Figure 1A**), implying participation of RbbA with an IM protein, YhjD.

**Figure 1:** Analysis of RbbA and YhjD purifications and Localization on 30S ribosomes. (A) Immunoblot analysis of the indicated His_6_-RbbA (panel II) or YhjD (panel III) fusion protein in whole cell lysates (WCL) and anti-FLAG immunoprecipitates (IP) from an untagged DY330 strain and *E. coli* expressing a SPA-tagged YhjD or 30S r-subunits. Expression of affinity-tagged proteins from 30S r-subunits and YhjD in whole cell lysates (panel I) is monitored using M2 anti-FLAG antibody; molecular masses (kDa) by SDS-PAGE are indicated. The unrelated SPA-tagged YchM strain served as control. (B) RbbA and YhjD purifications showing common co-purifying proteins involved in 30S r-subunits, protein synthesis and in membrane processes. The co-purifying proteins were detected in two out of three different detergents tested. Yellow nodes represent the tagged bait proteins. Red edge reflects the *E. coli* proteins as “preys” interacting with RbbA and YhjD. Prey represented with similar node color is grouped according to COG (Clusters of Orthologus Group) functional categories. (C) Fractions from sucrose density gradient of ribosomes from affinity-tagged RbbA and YhjD strains were immunoprecipitated and analyzed by immunoblot using anti-FLAG antibody as described in Figure 1A. The signals detected from each fraction by immunoblot were quantified and are shown at the bottom of Panel C.

We then examined the proteins that co-purified with both RbbA and YhjD in at least two different detergents. Proteins that are involved in membrane (e.g. Trg, LolB, LptD, PhoS and KefA) and 30S (e.g. RpsN, RpsM, RpsS, RpsT, RpsP and RpsE) subunit r-proteins were consistently and reproducibly co-purified with RbbA and YhjD affinity tagged proteins (**Figure 1B**). Association of RbbA and YhjD with r-proteins of 30S (RpsN, RpsM, RpsS, RpsT and RpsE) subunits were additionally confirmed by immunoprecipitation, where ectopically expressed His_6_-tagged RbbA co-precipitated from detergent extracts containing the affinity-tagged 30S subunit r-proteins (**Figure 1A**). Since the tagged RbbA and YhjD interacted with 30S subunit r-proteins, we also examined their binding site on the fully assembled 70S ribosomes and its subunits isolated through sucrose density gradients using anti-FLAG M2 monoclonal antibody. As shown in **Figure 1C**, both RbbA and YhjD localize to the 30S subunit. Even after prolonged exposure, cross-reactivity was observed only on the 30S subunit. These and the physical interaction results indicate that RbbA and YhjD indeed bind to 30S subunits.

RETRACTED

Apart from the 30S subunit r-proteins, the endogenous affinity-tagged YhjD co-purified strongly with certain energy regeneration and membrane ABC Transporter pathway components (**see Text S2**) including an outer membrane (OM; LptD) and with two IM (LptB and MsbA) LPS transporters in the detergent extracts (**Table S1)**. The later observation is consistent with the recent implication on the function of YhjD protein in LPS transport [11], [12]. Conversely, the affinity-tagged RbbA bound only to the LptD protein in detergent extracts. Although the mass spectrometry failed to detect the two other LPS components with RbbA, we were able to confirm these associations, including LptD by immunoprecipitation from cell-lysates derived from strains containing C-terminal affinity-tagged MsbA, LptB and LptD proteins (**Figure 2A**). Thus, the stable association of these two affinity-tagged proteins with LPS transport components suggests the possibility that they might cooperate with LPS proteins to mobilize phospholipids and alter the fluidity of the membrane by providing a mechanism to move LPS molecules into and/or across the OM barrier.

**Figure 2:** Localization of RbbA and YhjD on membranes. (A) Immunoblot analysis of the indicated His_6_-RbbA fusion protein in whole cell lysates (WCL, panel II) and anti-FLAG immunoprecipitates (IP, panel II) from an untagged DY330 strain and *E. coli* expressing a SPA-tagged MsbA, LptB and LptD proteins. Expression of affinity-tagged proteins from MsbA, LptB and LptD in cell lysates (panel I) is monitored using M2 anti-FLAG antibody. The unrelated SPA-tagged YchM strain served as control. Molecular masses are shown in kDa. (B) Intracellular localization of RbbA-YFP and YhjD-YFP using MinD-YFP fusion as control. Arrows show the YFP localization at the cell poles (top panel). Percentage YFP cells in one or two ends of the cell poles (bottom panel) for the indicated YFP-strain is an average of at least four experiments. Error bars indicate mean ± SD. Scale bar equals 2 µm. (C) Differential interference contrast images of temperature induced changes of cell morphology and the average cell length of the *rbbA*-*yhjD* double mutant and their respective single mutants at indicated temperatures are shown on the right side of panel C. The *minD*Δ served as control. Scale bar equals 2 µm.

RETRACTED

### Intracellular Localization of RbbA and YhjD

The protein interaction data suggested a potential role for RbbA and YhjD in membrane processes. To find whether RbbA and YhjD localize to the membrane, we constructed C-terminal fusions of RbbA and YhjD to yellow fluorescent protein (YFP). A strain producing the YFP fusion to MinD was used as a control. MinD is an ATPase that, when bound to ATP, localizes peripherally to the cytoplasmic membrane at one end of the two cell poles [14], [15]. Similar fluorescence patterns were observed in the RbbA-YFP and YhjD-YFP strains with about 43% of the >200 cells analyzed showing a fluorescent zone at one end of the cell (**Figure 2B**). In addition, ∼13% of the cells had fluorescent zones at both poles, suggesting that RbbA and YhjD most likely associate with the cell membrane or possibly anchor to the membrane surface. The similarity in fluorescence patterns of RbbA and YhjD with a cell division protein suggests that RbbA and YhjD might also cross talk to cell division.

Since translation affects many aspects of cell division [16], the morphology of the cells was examined at different temperatures in the *rbbA*Δ and *yhjD*Δ mutants. As shown in **Figure 2C**, the *rbbA*Δ and *yhjD*Δ single mutants appear to be slightly elongated; with average cell length of the mutant cells (∼5.0±0.7 µm) being almost 0.8 fold than that of the wild type cells (from 4.1±0.4 µm to 3.4±0.4 µm) at both 15 and 32°C. Remarkably, the double mutant appears to be even more elongated at both 15 and 32°C, with average cell lengths ranging from ∼9.0±0.32 to 7.2±0.35 µm, and resembled the *minD* (∼11.3±1.49 to 9.9±0.98 µm) control mutant [17]. The phenotype of the double mutant is more evident at 15°C compared to other temperatures. At 44°C, the cells from these deletion strains appeared shortened, restricted in cell size and unviable. These data reconfirm the attachment of RbbA and YhjD to the membrane and imply a connection of these two genes in cell division and protein synthesis.

### Genetic Interactions Suggest Involvement of RbbA and YhjD in Energy Generation, Protein Synthesis and Cell Division

Since genetic interactions are an informative means to discover functional relationships among genes [18], we used a recently developed eSGA (*E. coli* Synthetic Genetic Array) approach [19] to identify *E. coli* genes that genetically interact with *rbbA* and *yhjD*. In this conjugation-based assay, we generated double mutants by conjugating *rbbA* or *yhjD* donor strain (marked with Δ*::*Cm^R^) with single gene deletions of almost all other non-essential *E. coli* genes as well as hypomorphic alleles of selected essential *E. coli* genes (recipients marked with *Δ::*Kan^R^) (**Table S2**). The colony growth and relative fitness of the resulting double mutants surviving dual drug selection was then examined by digital imaging. Using a statistical interaction score (*S*) to quantify both the strength and confidence of the interactions between each *E. coli* mutant gene pair, we detected cases of both aggravating (synthetic sick or lethal (SSL)) as well as alleviating (i.e. positive or suppressing) interactions. Two genes are said to have aggravating or alleviating genetic interactions when the double mutant grows significantly worse or better, respectively than expected based on the phenotypes of the corresponding single mutants [19]. Aggravating or alleviating genetic interactions suggest that the protein products of the two genes are functionally related and are usually interpreted in terms of redundancy (parallel pathways) or similarity (same pathway) of function, respectively [20].

RETRACTED

As for the protein interaction experiments, we also observed genetic interactions of *rbbA*Δ and *yhjD*Δ with deletions of several energy regeneration genes. These included SSL interactions with members of the ETC: NADH dehydrogenases (namely NDH-1 and NDH-II from complex I), succinate dehydrogenases (*sdhCDAB* from complex II), cytochrome *bo* terminal oxidase complex (*cyoABCD* from complex IV), ATP synthase (*atpAC* from complex V), iron-sulfur (Fe-S) cluster proteins and with a few other catabolic genes encoding enzymes which reduce the NDH pool and reduce the electron flux through the ETC (**Figure 3A** **, Table S2**). In addition, a synthetic sick interaction was observed between the *ΔrbbA* mutant as donor and *ΔyhjD* as recipient or vice-versa (**Table S2**). Over-representation analysis using GO annotation terms showed that the interacting genes identified in the *rbbA* and *yhjD* deletion screens were enriched significantly (q-value <0.05) for genes involved in the ETC, tricarboxylic acid cycle, ATP-synthesis coupled electron transport, lipid biosynthesis, fatty acid synthesis, rRNA and tRNA processing, as well as other processes linked to membrane, protein synthesis and energy metabolism (**Tables S3 and S4, see Text S3**).

RETRACTED

**Figure 3:** Functional redundancy of RbbA and YhjD with oxidative phosphorylation genes. (A) Diagrammatic representation of the ETC system of *E. coli* modeled based on [55]. The diagram shows the SSL interactions from *rbbA* and *yhjD* donor deletion strains with members of the pathway: Fe-S cluster, complex I, II, IV, V and some key genes encoding catabolic enzymes. The cytochrome *bc_1_* or cytochrome *c* oxidases of complex III does not occur in *E. coli* [56]. Q: ubiquinone; FMN: flavin mononucleotide; FAD: flavin adenine dinucleotide. Blue represents aggravating (negative *S* score) interaction. (B) Chromosomal positions of *rbbA* and *yhjD* (green arrows), individual gene deletions in *nuo* (complex I), *sdh* (complex II), and *cyo* (complex IV) operons (purple arrows), and other gene (red arrows) deletions used as donors (marked with Cm^R^) or recipients (marked with Kan^R^) in eSGA experiments are shown in the top panel. Other (*mdtF*, *malQ* and *dppC*) donor deletions (blue arrows) located close to the *rbbA* and *yhjD* genes served as controls for effects of proximity on recombination. Validation of *rbbA* and *yhjD* interactions and with energy producing pathway genes is shown in the bottom panel. The *rbbA*, *yhjD*, and control (*mdtF*, *malQ* and *dppC*) Hfr Cavalli donor deletion strains were crossed with the indicated F- recipient deletion strains, followed by selection on plates containing chloramphenicol and kanamycin.

The genetic interactions were re-examined in more detail to confirm some of the whole genome deletion screen results of *ΔrbbA* and *ΔyhjD* with the ETC pathway and to confirm the interaction of *rbbA* with *yhjD* or vice-versa. Thus, we individually deleted 8 of the 13 *nuo*-subunits of NDH1 (e.g., *nuoA, nuoB*, *nuoF, nuoJ, nuoK, nuoG*, *nuoL* and *nuoN*) from complex 1, 4 of the *sdh*-subunit genes of succinate dehydrogenases (s*dhCDAB*) from complex II, and 4 of the 4 *cyo*-subunit genes of *bo* terminal oxidase from complex IV (*cyoABCD*) and conjugated the resulting F^-^ recipients with *ΔrbbA* and *ΔyhjD* donor mutants (**Figure 3B**). Consistent with our *rbbA* and *yhjD* whole genome deletion screens, the recipient NDH1 and *sdh* complexes bearing individual gene deletions exhibited SSL phenotypes when combined with *ΔrbbA* and *ΔyhjD* donor mutants. Accordingly, the *ΔrbbA* mutant exhibits a SSL phenotype with members of complex IV of the ETC. Conversely, no apparent effect on growth was observed with the *ΔyhjD* donor and the recipient electron transport complex IV mutants. However, there was a slight growth defect consistently apparent between the *ΔyhjD* donor and the *ΔcyoA* and *ΔcyoD* recipient mutants (**Figure 3B**). In addition, the *ΔyhjD* recipient and the *ΔrbbA* donor mutant or vice-versa, exhibited a significant synthetic sick growth defect (**Figure 3B**). We also confirmed that these observed genetic interactions were not a consequence of recombinant suppression resulting from gene proximity because no noticeable effects on growth were observed when *ΔrbbA* or *ΔyhjD* donor mutants were combined with deletions of functionally unrelated genes flanking *nuo*, *sdh* and *cyo* operons. Moreover, the use as donors of other unrelated genes in the same region, namely *mdtF*, *dppC* and *malQ* did not reveal synthetic genetic interactions with *rbbA* or *yhjD* (**Figure 3B**). Thus, RbbA and YhjD may not only appear to function redundantly among themselves but also with genes involved in part of the energy generating systems.

RETRACTED

The *rbbA*Δ and *yhjD*Δ eSGA screens also identified SSL interactions with cell division inhibitors, *minC* and *dicB*. MinC together with DicB appear to provide specificity for the septal rings in *E. coli* [21]. The SSL interactions were also observed with genes involved in cytoplasmic membrane-bound sensory histidine kinases (e.g., *rcsB*, *narQ*, *narX*, *rstB, envZ*, *cuss*, *cheA* and *torS*), phosphotransfer (e.g., rcsC) and DNA-binding two-component regulatory system (e.g., *rcsC*, *ompR* and *phoB*), the key mediators of the cellular response that senses cell envelope stress and in transduction of signals that enable cells to respond and adapt to their changing environments [22]. Genes involved in protein synthesis such as EF-Tu (*tufB*), 30S ribosomal subunit proteins [e.g., rpsF (S6), rpsU (S21) and rpsO (S15)] also showed SSL interactions with both *rbbA* and *yhjD* donor mutants. Thus, like the physical interaction and YFP localization data, the genetic interaction data not only suggest functional links between RbbA and YhjD in oxidative phosphorylation, but also points to the participation of RbbA and YhjD in signal transduction, protein synthesis and cell division.

### RbbA and YhjD Mutants Impair Translational Fidelity *In Vivo*

Since RbbA and YhjD physically interact with r-proteins, we further assessed their possible function in protein synthesis by comparing the [^35^S]-methionine incorporation into total proteins for the *rbbA*-*yhjD* double mutant and the corresponding single mutants to wild type cells at 32°C for 30 min. The total protein synthesized in the *rbbA*-*yhjD* double mutant was significantly lower than that observed with each single mutant, and was also significantly lower than the wild type (**Figure 4A**). Thus, the coordinate behavior of *rbbA* and *yhjD* suggests that both genes affect translation in a manner reminiscent of genes that suppress common functions.

RETRACTED

**Figure 4:** Protein synthesis, miscoding and ETC are impaired by deletions of *rbbA* and *yhjD*. (A) Incorporation of [^35^S]-methionine into total proteins of the wild type and the indicated deletion strains in the absence and presence of sodium azide (500 µM) or CCCP (10 µM). Error bars indicate mean ± SD. (B) Elevated rates of frame-shifting and stop-codon read-through in wild type and in the indicated deletion strains in the absence and presence of sodium azide (500 µM) or CCCP (10 µM). Error bars indicate mean ± SD. The β-gal activity is normalized to the activity of β-lactamase that has been used as an internal control. (C) Immunoblot of the full-length and truncated β-gal is assayed after transforming the reporter plasmid pSG400 carrying a premature UAG stop codon expressed in *rbbA-yhjD* double mutant (Lane 4) and in the *rbbA* (Lane 2) and *yhjD* (Lane 3) single mutants. The assay was also performed with another reporter plasmid 4pCCCU containing +1 frame-shift expressed in *rbbA*-*yhjD* double mutant (Lane 8) and in the *rbbA* (Lane 6) and *yhjD* (Lane 7) single mutants. The wild type and plasmids pSG400 (Lane 1) and 4pCCCU (Lane 5) served as controls. (D) Growth sensitivity assay of the indicated deletion strains in the presence or absence of antibiotics affecting miscoding, translocation and accuracy of protein synthesis. The minimum inhibitory concentration (MIC) of the antibiotic is shown in parenthesis. The hypomorphic allele of the essential gene *fusA* and the non-essential mutant *tufB* served as controls. (E) Serial-dilution assay showing the reduced growth fitness defect of *rbbA*-*yhjD* double mutants and their corresponding single mutants on M9 minimal media in the presence of 2% glucose or glycerol. (F) Growth sensitivity of the indicated deletion strains in the presence or absence of piericidin A targeting the NDH (Complex I) in ETC. The MIC of the drug is shown in parenthesis. The *nuoL* mutant served as control.

Because the *rbbA* and *yhjD* mutants appeared defective in the synthesis of proteins (**Figure 4A**), we assessed the translational fidelity of the mutants *in vivo* by examining the expression of full-length β-galactosidase (β-gal) from a template harboring out-of-phase nonsense codons in its coding sequence. As shown in **Figure 4B**, compared to the wild type, the *rbbA* and *yhjD* mutants did not exhibit significant read-through of either the amber (UAG) or the opal (UGA) mutants of β-gal. However, the *rbbA*-*yhjD* double mutant exhibited higher read-through of both UAG and UGA β-gal mutants. Western-blot analysis of the cell lysates from the single and double gene deletions transformed with the two different reporter plasmids verified the expected presence of the truncated β-gal specified by the UAG or +1 frame-shift mutations. However, the full-length β-gal is synthesized significantly only by the double mutant, which also encoded correspondingly less of the truncated protein (**Figure 4C**). Thus, it appears that nonsense codons are indeed mistranslated in the double mutant. Further study of β-gal +1 and -1 frame-shift mutations revealed that, relative to the wild type, the single mutants were only slightly affected while the double mutant exhibited significantly higher miscoding of both +1 and -1 frame-shift mutations in β-gal. These results suggest that the double mutant has significant lesions in translational miscoding.

RETRACTED

If *rbbA* and *yhjD* mutants display a significant loss of translation fidelity, then the cells carrying deletions of *rbbA* and *yhjD* should display enhanced sensitivity to antibiotics that interact with ribosomes and promote translational errors. Thus, we compared the sensitivity of the *rbbA* and *yhjD* single and double mutants and of the wild type to antibiotics affecting decoding by the 30S subunit (e.g., streptomycin, neomycin and paromomycin). Tetracycline targeting the ribosomal A-site [23], fusidic acid hampering translocation and ribosome recycling [24], [25], and streptomycin fostering miscoding of near-cognate aminoacyl-tRNAs [26] had a very small effect on the growth of the deletion strains (**Figures S2A and S2B**). Conversely, all the mutants appear sensitive to paromomycin implying an altered miscoding of sense codons [27] (**Figure 4D**). However, the deletion mutants were relatively resistant to the aminoglycoside antibiotic neomycin, which alters miscoding (**Figure S2B**), whereas other aminoglycosides, i.e. gentamycin and spectinomycin, known to impair translocation and accuracy of tRNA ejection during proof-reading [27], markedly interfered with the growth of the deletion strains (**Figure 4D**). The sensitivity of the *rbbA*-*yhjD* double mutant to the same spectrum of antibiotics strengthens the connection of these genes to the translation process. In the same experiment, the hypomorphic allele of the essential gene *fusA* and the non-essential *tufB* mutant were used as controls. The *tufB* mutant was expected to grow because the cell carries an identical gene *tufA*. The *fusA* gene encoding EF-G, which enables translocation, was affected to varying degrees by all the antibiotics tested [28]. This may reflect the fact that EF-G alters not only translocation but also ribosome recycling, a process that requires the ribosome recycling factor (RRF), elongation factor G (EF-G) and release factor (RF-3) [24], [25], [29]. Indeed, the residual translation observed in the absence of the *fusA* gene is targeted by antibiotics reported to alter spontaneous translocation artificially induced by treatment of ribosomes with dithiol-specific reagents [27]. The resistance of *rbbA*Δ or *yhjD*Δ mutants to antibiotics was restored to wild type levels by expression of RbbA or YhjD (**Figure 4D**; only *rbbA* complementation is shown). Thus, it appears that the fidelity of translation may be impaired by *rbbA* and *yhjD* mutations. It seems particularly significant that the *rbbA*-*yhjD* double mutant increased the sensitivity of *E. coli* to antibiotics to a level comparable to that of the *rbbA* and *yhjD* single gene deletion strains, implying that these proteins may be part of a singular pathway. Furthermore, the lack of additive sensitivity phenotype between the *rbbA* and *yhjD* mutations suggests that there may be a functional overlap between *rbbA* and *yhjD* where one gene compensates for the absence of the other.

RETRACTED

### Inhibition of Electron Transport Impairs RbbA and YhjD Functions as well as Protein Synthesis and Translational Fidelity

The genetic interactions of RbbA and YhjD suggested a functional relation to oxidative phosphorylation. This was also suggested by the finding that the single and double mutants grew poorly in glycerol media compared to glucose implying that they were compromised in aerobic respiration (**Figure 4E**). To verify the functional linkage of these proteins with the ETC we blocked the electron flow of the oxidative phosphorylation chain using piericidin A, a selective inhibitor of NDH (Complex I) [30] where 90% of the membrane potential due to the redox reaction of complex I activity has previously been shown to be inhibited in *E. coli* [31], [32]. Remarkably, piericidin A inhibited the growth of *rbbA*-*yhjD* double mutant in the whole cell extract to the same extent as their single mutants (**Figure 4F**). The observed phenotype is indeed caused by deleting *rbbA* or *yhjD* because a pBAD-plasmid expressing RbbA or YhjD under the control of an arabinose-inducible promoter, but not a control plasmid without the respective genes, restored the antibiotic resistance of *rbbA* or *yhjD* null strains to wild type levels (**Figure 4F**; only *rbbA* complementation is shown). Thus, it appears that the growth phenotype observed with the *rbbA-yhjD* double mutant and their respective single mutants may be linked to the electron transport pathway.

To verify the functional linkage between protein synthesis and the ETC, we challenged the *rbbA*-*yhjD* double mutant and their respective single mutants with CCCP (carbonylcyanide-m-chlorophenylhydrazone), a proton-ionophore which not only diffuses across the IM and the periplasmic space in the protonated form [33] but also rapidly dissipates the proton motive force [34]. In parallel, the mutants were also treated with sodium azide, a respiratory chain inhibitor depolarizing the bacterial cell membrane [35], which blocks the ATP hydrolysis that is coupled to protein translocation [36]. As shown in **Figure 4A**, CCCP or azide, used at sub-inhibitory concentrations, markedly reduced the incorporation of [^35^S]-methionine into total proteins of the cells harboring the *rbbA*-*yhjD* double mutant and their respective single mutants, implicating that these agents disrupt the ETC markedly by interfering with the protein synthesis as expected. Surprisingly, the single mutants in the presence of azide or CCCP showed a negligible increase in β-gal synthesis compared to the single mutants in the absence of the drugs (**Figure 4B**). On the other hand, the double mutants exhibited significantly more -1 and +1 frame-shift errors as well as UAG and UGA nonsense codon read-through in the presence of azide or CCCP (**Figure 4B**). Although these results suggest that perturbation of the ETC impairs translational fidelity resulting in enhanced translational miscoding and frame-shift errors in β-gal, there is an unquestionable functional connection between the action of RbbA and YhjD that links the process of protein synthesis to energy generating processes harbored by the membrane and specifically to the ETC.

RETRACTED

## Discussion

The ribosome-dependent ATPase elongation factor, RbbA, belongs to a large class of ABC ATPases that act in a variety of small molecule transport mechanisms as well as in protein synthesis [37], [38]. The closest functional and structural homologue of RbbA is elongation factor EF-3 of *Saccharomyces cerevisiae* which shares a common function in translation and several sequence motifs such as an ELVES motif present in tRNA binding proteins, two “LSGGQ” ATP binding motifs and two Walker motifs (ABC cassettes) that define this ABC class of transporters as the most abundant ATPases in all cells [38]. The folding patterns of the two proteins reveal a striking similarity in domains I-II in RbbA and domains II-III in EF-3, underlying their structure and strengthening the connection between RbbA and EF-3 (**Figure S3A and S3B**). There are, however, features which differ in the sequences of these proteins. The N-terminus of EF-3 has a HEAT domain which is absent in RbbA (**Figure S3B**) and was shown by Cryo-EM analysis to bind to the head of the 80S and reach the L1 stalk of the yeast 60S ribosomal subunit E-site, suggesting that it may participate in release of deacyl-tRNA from ribosomes during each step of elongation [39]. Although RbbA lacks the HEAT domain, it interacts directly with the E-site and has been shown to accelerate release of deacyl-tRNA from ribosomes during protein chain elongation [1]. The C-terminus of EF-3 is a stretch of dispensable basic amino acids. In contrast, RbbA has six predicted transmembrane helices (residues 563-906 of the 911 amino acids) at its C-terminus, pointing to its potential to interact with membranes. Although these features suggest a dual localization of RbbA on ribosomes and on membranes, the cellular role of RbbA is yet not fully understood. Here, we use biochemical and genetic approaches to examine the possible connection of RbbA to protein synthesis, membrane processes and energy sources.

RETRACTED

The physical interaction study we report shows that RbbA binds to the membrane and reciprocally co-purifies with an IM protein of unknown function, YhjD, implicated in LPS export across the IM [12]. Mutations based on single amino acid substitutions in either MsbA, an IM, essential ABC transporter in the LPS export pathway or in YhjD suppress the lethal consequence of an incomplete lipid A precursor IV_A_ [11]. However, the physical evidence we report shows that RbbA, as well as YhjD, co-purifies with other members of the LPS export pathway (i.e. MsbA, LptB and LptD), suggesting that RbbA and YhjD, together with an as-yet-unidentified transmembrane partner, may form a membrane-associated complex with LPS proteins and thus both proteins are likely to have a role in LPS transport across the IM. Remarkably, both proteins interact with the same 30S ribosomal subunit proteins, with a related number of ABC transporters, and with proteins that are integral to the *E. coli* membrane (**Table S1**).

Alterations in membrane composition due to mutations have effects upon membrane protein folding, electron transport, initiation of DNA replication, protein synthesis and cell division [40]. Consistent with this notion, the genome wide genetic screen of the *rbbA* mutant displayed a SSL interaction with *yhjD* and with members of complexes I, II and IV of the ETC. Phospholipids that reside in the membrane are vital to the function of the proton gradients responsible for the synthesis of ATP by the ETC *via* ATP synthase. In fact, disruption of phospholipids of the ETC is expected to impair the proton gradient, thus inactivating the synthesis of ATP [41]. Thus, the SSL phenotype of the ETC imparted by deletion of the *rbbA* and *yhjD* genes can be partly explained by the effect of these proteins on phospholipids of the ETC. Our observations from the genetic interactions complement the biochemical results demonstrating that RbbA is functionally an important component of the membrane bound YhjD. The regeneration of the active or ATP form of *rbbA* may occur by virtue of its proximity to the *yhjD* membrane protein and in turn to the ETC. Interestingly, phospholipids are known to accelerate the rate of ATP:ADP exchange [42] supporting the suggestion that the attachment of RbbA to the membranes may indeed enhance its ability to exchange bound ADP to the active bound ATP form which is needed for protein synthesis.

RETRACTED

Moreover, RbbA and YhjD also appear to affect cell division. The similarity in the YFP localization patterns of RbbA and YhjD with a MinD cell division protein reconfirmed the attachment of these proteins to the membrane as well their role in cell division. The *minD* mutants apparently allow polar divisions because of their affinity for the phospholipid tubes which occur at the cell poles, and restrict the potential for division to mid cell [43]. The observation that RbbA and YhjD physically bind to LPS proteins and exhibit a similar cell division phenotype as MinD may also be explained by alterations in phospholipids. In fact, the conversion of membrane bound MinD•ADP to the active MinD•ATP occurs in a phospholipid dependent fashion [44]. The appearance of more elongated cells in the RbbA and YhjD double mutant under permissive growth conditions (i.e. at 15°C and 30°C), also suggest a role for these proteins in cell division. It is important to restate that the appearance of an elongated phenotype in the double mutant is not just an artifact of cell death taking place at lower or at normal growth temperatures. Thus, it is likely that RbbA and YhjD play redundant roles in membrane biology necessary for the completion of cell division. A role of RbbA and YhjD in cell division is also suggested by its aggravating genetic interactions with various known cell division factors (e.g., *minC, dicB*). Another explanation for the possible involvement of these two proteins in cell division is that the ATP supply might be lower prior to division events, leading to curtailment of replication and protein synthesis. Such a phenomenon takes place in eukaryotic cells where the amount of ATP is greatly reduced in the G1 phase of the growth which precedes cell division [45]. In some cases, new protein synthesis might also be required prior to the onset of DNA replication which precedes cell division [46]. Since total protein synthesis is greatly reduced in the *rbbA*-*yhjD* double mutant at 32°C (**Figure 4A**), it is possible that the impaired cell division observed in the double mutant is due to limitation of certain proteins needed for DNA replication prior to the cell division. Curiously, the ability of RbbA to promote cell division at 15 and 32°C, appears to function in cooperation with the ETC and requires a functional YhjD.

RETRACTED

Apart from their role in membrane biogenesis, the presence of an RNA binding motif inscribed in both RbbA and YhjD sequences as well as the reciprocal physical interaction of these proteins suggested that like RbbA, YhjD may also function in protein synthesis. Our physical evidence indicates that these two proteins localize to the 30S ribosomal subunits. Further, the *rbbA* and *yhjD* double mutant and their respective single mutant cells showed comparable level of sensitivity to antibiotics targeting translational fidelity. This suggests that YhjD indeed functions in protein synthesis in cooperation with RbbA. *In vitro* studies on RbbA suggest a role in synthesis accuracy as it restricts miscoding of amino acids and since paromomycin, an antibiotic which interferes with translational fidelity, antagonizes the RbbA-dependent synthesis (data not shown). These *in vitro* experiments also suggest that the reduction of miscoding by RbbA is due in part to its interaction with EF-Tu. Indeed this pairwise interaction between RbbA and EF-Tu (e.g. TufA, TufB) is being detected by our mass spectrometry analyses (**Table S1**).

Exposure of the *rbbA*-*yhjD* double mutant cells to chemical agents that block the electron flow of the oxidative phosphorylation chain also severely restricted the incorporation of amino acids into proteins to a level comparable to each of the single mutants, implying once again a connection between RbbA and YhjD in protein synthesis and in the functioning of the ETC. However, it was surprising that the cells from the *rbbA*-*yhjD* double mutant exhibited an exaggerated increase in miscoding of β-gal synthesis which was not evident in the single mutants. These results suggest that there may be functions compensating for miscoding when there is loss-of -function in one of the alleles but such compensatory mechanisms may not keep pace with the loss of both functions and thus result in an increased error rate observed with the double mutant. For example, it is entirely possible that EF-Tu, which is essential for the accuracy of protein synthesis and functions with RbbA, may suppress the loss of the *rbbA* gene. In turn, the *rbbA* gene might suppress some of the functions affected by loss of the *yhjD* gene. Another possibility is that the reduced ATP concentration may suffice to reduce the translational errors observed in the single mutants but may not adequately compensate for the miscoding events observed when these errors are compounded in the double mutant. In any case, the decrease in the cellular supply of ATP derived from the ETC is expected to exacerbate at least some of the translation and fidelity defects observed with the mutants reported here.

RETRACTED

We consider the possible repercussions of the effects of these proteins on membrane and protein synthesis processes. First, these proteins might alter the biosynthesis of several integral membrane proteins by membrane bound ribosomes, which requires their insertion into a phospholipid bilayer, a process governed by membrane-bound transporters which facilitate threading of appropriate polypeptides through the membrane [47], [48]. Second, it is possible that RbbA and YhjD act as chaperones during membrane synthesis and/or assembly. Thus, it is conceivable that the localization of these proteins on ribosomes and on membranes may be used to transport LPS through membranes, thus creating conformational changes in the membrane that are transmitted to ribosomes. The attachment of ribosomes to membranes in the process of protein secretion and during membrane biogenesis is well known [48] but possible connectivity between OM signals and the translation process have not been described. Nonetheless, it may be that the heterogeneity of ribosomes implicated as a regulatory feature of the particles [49] is used to bind ribosomes to specific IM sites that are involved in the formation of respiratory chain complexes, ribosome biogenesis and/or sensors that transmit extracellular stimuli from ribosomes to the translation machinery. Such an attachment of ribosomes to the IM may occur at discreet sites on the membrane to insure the entry of proteins in a defined orientation for proper assembly of membrane structures.

The evidence we present implicates a direct association of RbbA and YhjD through physical and genetic interactions as well as through the common membrane and ribosome targets. We suggest that the association of these proteins, however disparate be their detailed mechanism, is part of a cellular link between the energy requirement in protein synthesis and the energy supplied by oxidative phosphorylation. It seems entirely possible that these proteins are part of a network of interacting pathways that connect external stimuli from the membrane to protein synthesis and possibly mediate regulation of growth and cell division. It is necessary for the cell to commit to diverse functions in compliance with its energy supply. Thus, the linkage of protein synthesis to the ATP supplied by the ETC may be essential to cellular survival. The finding that RbbA and YhjD are genetically and physically linked to the ETC in the cell points such a functional relationship.

RETRACTED

## Materials and Methods

### Bacterial Strains and Growth Conditions

The wild type and deletion strains used in this study are listed in **Table S5**. Deletion strains were from the Keio knock-out library [50]. Hfr donor strains were constructed using λ-Red recombination [19]. Media and plates were supplemented with chloramphenicol (Cm, 34 µg/ml), kanamycin (Kan, 50 µg/ml), ampicillin (100 µg/ml), as required.

### Tagging and Purification

The endogenous RbbA and YhjD were C-terminally tagged using a sequential peptide affinity (SPA) dual tagging system and purified essentially as previously described [51], except in all purification steps 1% Triton or DDM or C12E8 mild non-ionic detergents were added to disrupt the association of RbbA with membrane fraction. The analysis of mass spectrometry data was essentially as previously described [51].

### Immunoprecipitation

In the case of overproduced His_6_-tagging and purification, the *E. coli* open reading frames cloned into a high copy pCA24N plasmid [52] with a chloramphenicol selectable marker was used to express C-terminal His_6_ - tagged fusion protein under the control of an IPTG inducible promoter. After 3 hrs induction at 30°C to an OD of ∼0.6, cells were harvested and lysed by sonication and the bait proteins purified by affinity chromatography under non-denaturing conditions essentially as previously described [51]. Immunoblots were performed essentially as previously described [51] with antiserum against FLAG and His epitopes.

### Yellow Fluorescent Protein and Cell Morphology Studies

C-terminal fusions of chromosomal RbbA, YhjD and MinD YFP strains were constructed in DY330 background by efficiently converting the respective *E. coli* SPA-tagged strains via λ-RED recombination system [51]. Briefly, PCR amplification was performed on an YFP-Cm resistance cassette (gift from Paul Choi and Sunney Xie, Harvard University) as a template. The PCR was performed using ∼40 bp primers homology to the insertion site (SPA) and ∼20 bp annealing to Cm resistance cassette. The YFP-fusion strains were grown exponentially in LB medium at 32°C. For cell morphological studies, the overnight deletion strain cultures on LB medium were sub-cultured and grown until the A_600_ value of the culture reaches 0.5. Prior to imaging, the cultures were incubated for 60 min at 15, 32 and 44°C. When required, images were captured using the Quorum WaveFX Spinning Disc Confocal System; cell length was measured using the Volocity program.

### Sucrose Gradient Centrifugation

The crude S30 extracts were loaded on linear sucrose density gradients as described [53], and 47% sucrose was used as cushion and ribosomes or subunits were sedimented at 4°C for 5 hrs.

RETRACTED

### Genome-wide eSGA Screens

A full-genome eSGA screen using *rbbA*Δ::Cm^R^ and *yhjD*Δ::Cm^R^ in Hfr Cavalli as donor was carried out and analyzed as previously described [19], as were with various mini-array crosses. Interaction scores (*S*) were calculated as previously described [19] to quantify the strength and confidence of the genetic interaction for each mutant gene pair. Gene set enrichment analysis was performed on the interaction *S* scores to determine the significant functionally related gene sets for GO terms spanning various biological processes (**see Text S3**).

### *In Vivo* Assays on Respiratory Competence and on Fidelity and Translocation

Growth of the *E. coli* wild type and deletion strains under starvation conditions were assessed by growing the cultures exponentially in LB media. The exponential phased cultures were serially diluted and plated onto M9 minimal media plates supplemented with 2% glucose or glycerol. For the drug sensitivity assays, exponentially growing wild type and deletion strains in LB medium were serially diluted and pinned onto LB plates in the absence or presence of the indicated concentrations of the antibiotics targeting the ETC or fidelity and translocation. Plates were incubated for 48 hrs at 32°C before scoring for any growth defects.

### Incorporation of Amino acids into Protein and Frame-shift Mutations of *rbbA* and *yhjD* Deleted Strains

The *E. coli* wild type and deletion strains were grown logarithmically in M9 minimal media without methionine. When the A_600_ value of the cultures reached 0.3, 10 µCi of [^35^S] methionine was incorporated into the growing cells. The translation reactions were incubated at 32°C and samples were drawn at 30 min. The rate of protein synthesis was determined as described previously [13]. Translation fidelity assay on the deletion strains were performed essentially as described [13] using previously reported expression plasmids [54], with the following modifications. Briefly, the *E. coli* cells were grown at 30°C to OD_600_ 0.4–0.6. Cell pellets were resuspended in 0.1 M phosphate buffer pH 7.5 and lysed by sonication. β-galactosidase assays were performed using the O-nitrophenyl-α-D-galactopyranoside (ONPG) method and the β-lactamase activities were measured using a CENTA kit (Calbiochem). The activity of β-galactosidase was normalized to that of β-lactamase.

The full-length and truncated β-gal activity in the deletion strains transformed with reporter plasmids were assessed by Western blotting using standard methodology. Briefly, 8 µg of the *E. coli* lysate from the deleted strains or the wild type was separated on 10% SDS/PAGE, transferred onto nitrocellulose membrane [51] and the β-gal activity visualized by probing the membrane against the rabbit anti-β-gal polyclonal antibody (Millipore^TM^). Each experiment was repeated independently at least six times. Incorporation of [^35^S]-methionine into total proteins and β-gal activity in the wild type and in the deletion strains treated with specific ETC inhibitors (sodium azide or CCCP) of ETC was assessed in the same manner as described above.

RETRACTED

## Supporting Information

Figure S1 **Comparative Sequence Alignments of RbbA and YhjD.** Amino acid sequence alignments of *E. coli* RbbA and YhjD proteins were determined by the CLC sequence viewer program. The RNA binding and two ATP binding (ATP-1 and ATP-2) motifs shared by the amino acid sequence of YhjD and RbbA are boxed in blue. The letters in red indicate the conserved amino acids.
(EPS)

Figure S2 **RbbA and YhjD show Reduced Protein Synthesis and their Growth is Perturbed with Antibiotics Targeting Fidelity and Translocation.** (A, B) Serial-dilution assay showing the perturbed growth of *rbbA*-*yhjD* double mutant and their corresponding single mutants in the presence of antibiotics targeting ribosomal A-site, translocation and ribosome recycling (Panel A) and in the presence of aminoglycosides targeting fidelity and decoding process of protein synthesis (Panel B) (see main text for details). The MIC of the antibiotics is shown in parenthesis. The controls were same as in Figure 4D.
(EPS)

Figure S3 **Comparative sequence alignments and folding patterns of RbbA and EF3.** (A) Amino acid sequence alignments of *E. coli* RbbA and *S. cerevisiae* EF-3 proteins were determined by the CLC sequence viewer ver 6.0 program. The two common Walker ATP binding motifs (ATP-1 and ATP-2) are underlined in blue and the blue rectangular box shows the common t-RNA binding motif. The letters in red indicate the conserved amino acids. (B) The crystal structures of RbbA and EF-3 determined at 2.7 Å resolutions was modeled using the SWISS-PROT folding program. The model used to draft the folding pattern of RbbA is based on sequence homology and strict folding pattern similarity to the ABCE1 transporter of *Pyrococcus abyssi* [57]. The positions of the RNA and ATP binding motifs and the location of N- and C-terminus of the RbbA and the folding pattern of the N-terminal end of RbbA lacking the HEAT domain (residues 1 to 321) are shown on the left panel. The crystal structure of EF-3 shown in right panel represents the common ATP and RNA binding motifs as well as the HEAT domain (residues 1-321) at the N-terminus of the structure.
(EPS)

Table S1 Protein-protein interactions from endogenous affinity tagged RbbA and YhjD in the presence and absence of various detergents.
(XLS)

Table S2 Genetic Interaction Scores of Hfr *rbbA*Δ and *yhjD*Δ Donor Mutants Screened against the Recipient F- Keio Non-essential Single Gene Knock-Out Library and 149 Potential Hypomorphic Essential Genes.
(XLS)

Table S3 Over-representation Analysis using Gene Ontology Terms on the Genetic Interaction Score from *rbbA*Δ Genome-Wide Genetic Screen.
(XLS)

Table S4 Over-representation Analysis using Gene Ontology Terms on the Genetic Interaction Score from *yhjD*Δ Genome-Wide Genetic Screen.
(XLS)

Table S5 Bacterial Strains used in this Study.
(XLS)

Text S1 RbbA Associates with Proteins Involved in Protein Synthesis and Membrane Processes.
(DOC)

Text S2 ABC Transporters and Energy-Linked Pathway Proteins Co-purifies with YhjD.
(DOC)

Text S3 Over-representation Analysis using Gene Ontology Terms on the Genetic Interaction Score from *rbbA*Δ and *yhjD*Δ Genome-Wide Genetic Screens.
(DOC)
